The article "Down-regulation of microRNA-142-3p inhibits the aggressive phenotypes of rheumatoid arthritis fibroblast-like synoviocytes through inhibiting nuclear factor-κB signaling" was retracted in 2020. Reasons: manipulated images; duplicated images; concerns about the images.

# Down-regulation of microRNA-142-3p inhibits the aggressive phenotypes of rheumatoid arthritis fibroblast-like synoviocytes through inhibiting nuclear factor-κB signaling

**DOI:** 10.1042/BSR20190700

**Published:** 2019-07-08

**Authors:** Jianhong Qiang, Tingting Lv, Zhenbiao Wu, Xichao Yang

**Affiliations:** 1 Department of Traditional Chinese Medicine, Yan’An People’s Hospital, No. 57, Qilipu Street, Baota District, Yan’an City 716000, Shaanxi Province, China; 2 Department of Rheumatology and Immunology, The Second Affiliated Hospital of The Fourth Military Medical University, No. 569, Xinsi Road, Xi’an City 710038, Shaanxi Province, China; 3 Department of Clinical Immunology, The First Affiliated Hospital of The Fourth Military Medical University, No. 1, Changle East Road, Xi’an City 710032, Shaanxi Province, China

**Keywords:** Inflammation, MicroRNA-142-3p, Nuclear factor-kappa B, Proliferation, Tumor necrosis factor α

## Abstract

The present study aimed to investigate the regulatory roles of miR-142-3p on the aggressive phenotypes of rheumatoid arthritis (RA) human fibroblast-like synoviocytes (RA-HFLSs), and reveal the potential mechanisms relating with nuclear factor-κB (NF-κB) signaling. miR-142-3p expression was detected in RA synovial tissues and RA-HFLSs by quantitative real-time PCR (qRT-PCR) and Northern blot analysis. RA-HFLSs were transfected with miR-142-3p inhibitor and/or treated with 10 µg/l tumor necrosis factor α (TNF-α). The viability, colony formation, apoptosis, migration, invasion, and the levels of interleukin (IL)-6, and matrix metalloproteinase 3 (MMP-3) were detected. The mRNA expressions of B-cell lymphoma-2 (Bcl-2), Bax, Bad, IL-6, and MMP-3 were detected by qRT-PCR. Moreover, the expression of Bcl-2, IL-1 receptor-associated kinase 1 (IRAK1), Toll-like receptor 4 (TLR4), NF-κB p65, and phosphorylated NF-κB p65 (p-NF-κB p65) were detected by Western blot. The interaction between IRAK1 and miR-142-3p was identified by dual luciferase reporter gene assay. MiR-142-3p was up-regulated in RA synovial tissues and RA-HFLSs. TNF-α activated the aggressive phenotypes of RA-HFLSs, including enhanced proliferation, migration, invasion, and inflammation, and inhibited apoptosis. miR-142-3p inhibitor significantly decreased the cell viability, the number of cell clones, the migration rate, the number of invasive cells, the contents and expression of IL-6 and MMP-3, and increased the apoptosis rate and the expressions of Bax and Bad, and decreased Bcl-2 expression of TNF-α-treated RA-HFLSs. MiR-142-3p inhibitor significantly reversed TNF-α-induced up-regulation of IRAK1, TLR4, and p-NF-κB p65 in TNF-α-treated RA-HFLSs. Besides, IRAK1 was a target of miR-142-3p. The down-regulation of miR-142-3p inhibited the aggressive phenotypes of RA-HFLSs through inhibiting NF-κB signaling.

## Introduction

Rheumatoid arthritis (RA) is a common autoimmune disease that affects 0.5–1% of the population worldwide [1]. RA is characterized by chronic inflammation in synovial tissues, and accompanied with the symptoms of pain, swelling, and stiffness of the joints [2]. Since RA contributes the destruction of cartilage and bone, RA is considered as one of the most common causes of disability [3]. In clinic practice, the therapeutic strategies for RA mainly focus on the control of pain and inflammation, as well as the protection of joint damage [4]. With the increasing revelation of the molecular mechanisms involved in the pathogenesis of RA, molecular targeting therapy has become a promising therapeutic strategy for RA.

Tumor necrosis factor α (TNF-α) is a proinflammatory cytokine that plays a key role in the pathogenesis of RA [5]. Since activated TNF-α is closely associated with the inflammation of synovial tissues, anti-TNF-α has become a promising therapeutic target for RA [6]. Until now, drugs targeting TNF-α have been widely applied in the treatment of RA, such as adalimumab, etanercept and infliximab [7,8]. However, the long-term application of TNF-α antagonists may be accompanied with the risk of infection and malignancy [9,10]. Therefore, novel therapeutic strategies for RA with high efficiency and safety are urgently needed.

MicroRNAs (miRs) are a family of small non-coding RNAs that involved in the occurrence and development of RA [11]. Previous studies have been proved that some miRs are up-regulated in RA, such as miR-146 [12], −155 [13], −203 [14], −221 [15], and −126 [16], and some are down-regulated, such as miR-34a [17], −124a [18], −22 [19], and −188-5p [20]. These miRs exert diverse regulatory roles in the aggressive phenotypes of RA human fibroblast-like synoviocytes (RA-HFLSs). For examples, miR-221 inhibitor inhibits the migration and invasion, and promotes the apoptosis of RA-HFLSs [15]. Lentivirus-miR-126 promotes the proliferation and inhibits the apoptosis of RA-HFLSs [16]. The precursor miR-124a suppresses the proliferation of RA-HFLSs by arresting the cell cycle at the G_1_ phase [21], and miR-188-5p mimic inhibits the migration of RA-HFLSs [20]. miR-142-3p is an important miR that involved in the regulation of inflammation [22,23]. It has been reported that miR-142-3p mimic alleviates bleomycin-induced apoptosis and overproduction of interleukin (IL)-1 and TNF-α in MLE-12 cells [22]. MiR-142-3p was down-regulated in the articular cartilage tissues of osteoarthritis (OA) mice, and the overexpression of miR-142-3p inhibits lipopolysaccharide (LSP)-induced apoptosis and the production of IL-1, IL-6, and TNF-α [24]. However, the specific regulatory roles of miR-142-3p on RA are still unclear.

In the present study, the expression of miR-142-3p was detected in both RA synovial tissues and RA-HFLSs. The regulatory effects of miR-142-3p on the aggressive phenotypes of RA-HFLSs, including the proliferation, apoptosis, migration, invasion, and inflammation were evaluated. In addition, the potential regulatory mechanisms of miR-142-3p related with nuclear factor-κB (NF-κB) signaling were further analyzed. Our findings may not only provide a novel therapeutic target for RA, but also reveal new insights into the underlying mechanisms of RA.

## Methods

### Patients

A total of ten RA patients (six males and four females, 52 ± 4 years old) were screened from our hospital between February 2017 and October 2017. During the same period, ten OA patients (three males and seven females, 52 ± 5 years old) were randomly screened. Both OA and RA were diagnosed according to the criteria established by the American College of Rheumatology. The present study was approved by the local Institutional Review Board, and informed consents were obtained from all subjects.

### Isolation and culturing of HFLSs

RA-HFLSs and OA-HFLSs were isolated from synovial tissues of RA and OA patients, respectively. Simply, synovial tissues were washed with phosphate buffer saline (PBS), cut into fragments, and digested with 0.1% Type-I collagenase (Sigma, St. Louis, MO, U.S.A.) for 4 h at 37°C. Followed by 5 min of centrifugation at 1000 rpm/min, HFLSs were resuspended in High-glucose Dulbecco’s modified eagle medium (H-DMEM) (Hyclone, Thermo Fisher Scientific, Waltham, MA, U.S.A.) containing 10% fetal bovine serum (FBS). Normal HFLSs, and HEK-293T cells (human renal epithelial cell line) were purchased from The Cell Bank of Chinese Academy of Sciences (Shanghai, China), and maintained in H-DMEM containing 10% FBS. All cells were cultured in a humidified incubator at 37°C with 5% CO_2_. The medium was refreshed every 2 days, and cells were passaged until 80–90% confluence. Logarithmic growth phase cells (third to eigth generation) were used for treatments.

### Cell transfection and treatments

MiR-142-3p inhibitor and miR-142-3p inhibitor negative control (INC) were purchased from Guangzhou Ruibo Biotechnology Co., Ltd. (Guangzhou, China). RA-HFLSs were seeded in 6-well plates at a density of 6×10^5^ cell/well, and transfected with miR-142-3p inhibitor or INC using lipofectamine 2000 (Thermo Fisher Scientific). After 24 h of transfection, the transfected-HFLSs were treated with 10 µg/l TNF-α for 24 h. RA-HFLSs were randomly divided into four groups, including Mock (RA-HFLSs without treatment), TNF-α (RA-HFLSs treated with TNF-α), INC + TNF-α (RA-HFLSs transfected with INC and treated with TNF-α), and Inhibitor + TNF-α (RA-HFLSs transfected with miR-142-3p inhibitor and treated with TNF-α).

### Quantitative real-time PCR

Total RNA was extracted from HFLSs using TRIzol agent (Thermo Fisher Scientific), and cDNA was reverse-transcribed using PrimeScript RT reagent Kit (TaKaRa, Japan) in accordance with manufacturer’s instructions. Quantitative real-time PCR (qRT-PCR) was performed on ABI 7500 (Applied Biosystems, Foster City, CA, U.S.A.) using specific primers (Table 1). The PCR program included 95°C for 3 min, 40 cycles at 95°C for 15 s, 60°C for 20 s, and 72°C for 20 s. U6 and GAPDH were used as internal controls. The relative expression of target genes were calculated according to the 2^−ΔΔ*C*^_t_ method [25].

**Table 1:** The sequences of specific primers used in qRT-PCR

Primers	Sequences	
	Forward	Reverse
miR-142-3p	5′-GGGTGTAGTGTTTCCTACT-3′	5′-CAGTGCGTGTCGTGGAGT-3′
U6	5′-TGCGGGTGCTCCGCTTCGGCAGC-3′	5′-CAGTGCAGGGTCCGAGGT-3′
IL-6	5′-TGTAGCATGGGCACCTC-3′	5′-CAGTGGACAGGTTTCTGAC-3′
Bcl-2	5′-GGTGGGGTCATGTGTGTGG-3′	5′-CGGTTCAGGTACTCAGTCATCC-3′
Bax	5′-AGGCCATCAGCAACAACATAAGT-3′	5′-GACAGCTTTGTGCTGGATCTGTG-3′
Bad	5′-AACTCGAGTGACAAGCCCGTA -3′	5′-GTACCACCAGTTGGTTGTCTTTGA -3′
MMP-3	5′-CGGTTCCGCCTGTCTCAAG-3′	5′-CGCCAAAAGTGCCTGTCTT -3′
IRAK1	5′-CCAAACATTGTGGACTTTGC-3′	5′-GGCTGTACCCAGAAGGATGT-3′
GAPDH	5′-TCCTCTGACTTCAACAGCGACAC-3′	5′-CACCCTGTTGCTGTAGCCAAATTC–3′

### Northern analysis of miRNAs

Northern analysis of miRNAs was performed as previously described [26]. Briefly, total 10 μg RNA was separated on 15% polyacrylamide–urea gels, transferred onto a Zeta-probe membrane (BioRad, Hercules, CA, U.S.A.) , and crosslinked by ultraviolet irradiation. The blots were pre-hybridized, and hybridized with specific probes, γ-32P end-labeled miR-142-3p probes or U6 at 37°C for 16 h.

### MTT assay

MTT was performed to detect the viability of RA-HFLSs. Simply, 200 μl RA-HFLSs were seeded in 96-well plates at a density of 6×10^3^ cells/well, and then incubated with 20 μg MTT (Sigma) for 4 h. After removing the medium, 150 μl DMSO was added into each well. Optical density (OD) at 495 nm was detected by a Microplate Reader (Molecular Devices, Sunnyvale, CA, U.S.A.).

### Colony formation assay

Colony formation assay was performed to detect the colony-forming ability of RA-HFLSs. Simply, RA-HFLSs were seeded in 6-well plates at a density of 500 cells/well, and cultured for 14 days. After removing the medium, the colonies were fixed in methanol for 15 min and stained with crystal violet for 15 min. The stained colonies were observed under microscope (Olympus, Tokyo, Japan), and counted by using the software of ImageJ version 1.48V (National Institutes of Health, Bethesda, MD, U.S.A.).

### TUNEL assay

TUNEL assay was performed to detect the apoptosis of RA-HFLSs. Simply, RA-HFLSs were fixed in 4% paraformaldehyde for 1 h, permeabilized with 0.1% TritonX-100/0.1% sodium citrate for 2 min, and blocked with 3% H_2_O_2_ for 10 min. Then cells were stained with TUNEL (Roche, Basel, Switzerland) in accordance with manufacturer’s instructions. Positive-stained cells were observed under microscope (Olympus), and counted in five randomly selected fields (×100).

### Wound healing assay

Wound healing assay was performed to detect the migratory ability of RA-HFLSs. Simply, RA-HFLSs were seeded in 6-well plates at a density of 5×10^5^ cells/well. When reaching 90% confluence, a wound track was scored in each well with a pipette tip. The cell debris were removed by washing with PBS. After 48 h of culturing, the migrated cells were observed under microscope (Olympus), and the migratory distance was measured.

### Transwell assay

Transwell assay was performed to detect the invasive ability of RA-HFLSs by using transwell chambers (BD, Franklin Lakes, NJ, U.S.A.). Simply, 100 µl cells were seeded in the upper chamber (pre-coated with Matrigel) at a density 1×10^5^ cells/well. The lower chamber is filled with 500 µl DMEM containing 10% FBS. Followed by 48 h of incubation at 37°C, cells on the upper chamber were removed with cotton swabs. Cells on the lower chamber were washed with PBS, fixed in 4% paraformaldehyde for 15 min, and stained with 0.1% crystal violet for 10 min. Positive-stained cells were observed under microscope (Olympus), and counted in five randomly selected fields (×100).

### Western blot

RA-HFLSs were lysed in RIPA Lysis buffer (Beyotime, Shanghai, China). Total proteins were separated by sodium dodecyl sulfate/polyacrylamide gel electrophoresis on 10% polyacrylamide gels, and transferred to polyvinylidenefluoride membrane (Millipore, Billerica, MA, U.S.A.). Then the membrane was blocked with 0.5% skim milk in Tris-buffered saline Tween (TBST) for 1 h, and incubated with specific primary antibodies (rabbit anti-human; anti-IRAK1, #ab245342; anti-TLR4, #ab13556; anti-p-NF-κB p65, #ab86299; anti-Bcl-2, #ab196495; anti-Bax, #ab32503; Bad, #ab32445; anti-GAPDH, #ab9485; 1: 1000, Abcam, Cambridge, England; NF-κB p65, 1:1000, #3033, Cell Signal, U.S.A.) overnight at 4°C. Followed by three times of washing with TBST, the membrane was incubated with horseradish peroxidase (HRP)-conjugated secondary antibody (goat anti-rabbit; 1: 5000, Sigma) for 1 h at 37°C. The protein brands were visualized using HRP color development kit (Thermo Fisher Scientific).

### Enzyme-linked immunosorbent assay

The contents of IL-6, and matrix metalloproteinase 3 (MMP-3) were detected in RA-HFLSs by using enzyme-linked immunosorbent assay (ELISA) kits (eBioscience, Thermo Fisher Scientific) in accordance with manufacturer’s instructions. The OD at 450/550 nm was measured by a Microplate Reader (Molecular Devices).

### Dual luciferase reporter gene assay

Dual luciferase reporter gene (DLR) assay was performed to identify the interaction between IL-1 receptor-associated kinase 1 (IRAK1) and miR-142-3p. Simply, HEK-293T cells were co-transfected with PsiCHECK-2 luciferase plasmids (Promega, Madison, WI, U.S.A.) carrying IRAK1-wild-type (PSMD11-WT)/IRAK1-mutant (PSMD11-MT) and miR-142-3p mimics/miR-142-3p mimics negative control (NC) (Ruibo). After 48 h of transfection, the fluorescence was visualized using a Dual Luciferase Reporter Assay Kit (Promega) according to the manufacturer’s instructions. The fluorescence intensity was detected by a Microplate Reader (Molecular Devices).

### Statistical analyses

All data were expressed as mean ± standard deviation. Statistical analysis was performed by SPSS version 18.0 (SPSS Inc., Chicago, IL, U.S.A.). Comparison between different groups was determined by *t* test (two groups) or one-way ANOVA (more than two groups). A *P* value less than 0.05 represented significantly different.

## Results

### MiR-142-3p was up-regulated in RA

The expression of miR-142-3p was detected in both RA tissues and RA-HFLSs. qRT-PCR showed that the expression of miR-142-3p in synovial tissues was significantly higher in RA patients than in OA patients, and was significantly higher in RA patients at stage IV than in those at stage III (*P*<0.05) (Figure 1A,B). RA- and OA-HFLSs were isolated from synovial tissues of RA and OA patients, respectively. The expression of miR-142-3p was significantly higher in RA-HFLSs than in OA-HFLSs (*P*<0.05). No significant difference on the expression of miR-142-3p was observed between OA-HFLSs and HFLSs (normal control) (Figure 1C). Additionally, Northern blot analysis showed that miR-142-3p was significantly up-regulated in RA patients compared with OA patients (Figure 1D). Similarly, expression of miR-142-3p in RA-HFLSs was higher than that in OA-HFLSs and TFLSs (Figure 1E).

**Figure 1:** The expression of miR-142-3p detected by qRT-PCR (**A**) Relative miR-142-3p mRNA expression in synovial tissues of OA and RA patients (*n*=10); (**B**) Relative miR-142-3p mRNA expression in synovial tissues of OA patients at stage III and IV (*n*=5); (**C**) Relative miR-142-3p mRNA expression in OA human fibroblast-like synoviocytes (OA-HFLSs), RA-HFLSs, and normal HFLSs; (**D**) Northern blot analysis of miR-142-3p in synovial tissues of OA and RA patients (*n*=10); (**E**) Northern blot analysis of miR-142-3p in OA-HFLSs, RA-HFLSs and normal HFLSs. *, *P*<0.05 versus OA (A) RAIII (B) or HFLS and OA-HFLS (C).

### Down-regulation of miR-142-3p inhibited TNF-α-induced proliferation of RA-HFLSs

The viability of RA-HFLSs was detected by MTT assay. As shown in Figure 2A, the viability (OD_495_ value) of RA-HFLSs was significantly increased with increasing concentrations of TNF-α in a dose-dependent manner until a peak at 10 µg/l (*P*<0.05). The results of Figure 2B showed the mRNA expression of miR-142-3p in inhibitor group was significantly decreased compared with Mock group and INC group (*P*<0.05), suggesting miR-142-3p inhibitor was successfully transfected. The treatment of 10 µg/l TNF-α significantly increased the viability of RA-HFLSs with increasing times in a time-dependent manner (*P*<0.05). The viability of RA-HFLSs was significantly higher in TNF-α group than in Mock group at different time points (*P*<0.05). In addition, the transfection of miR-142-3p inhibitor significantly decreased the viability of TNF-α-treated RA-HFLSs at different time points (*P*<0.05) (Figure 2C). Furthermore, colony formation assay showed that the number of cell clones was significantly higher in TNF-α group than in Mock group (*P*<0.05). The transfection of miR-142-3p inhibitor significantly decreased the number of cell clones formed by TNF-α-treated RA-HFLSs (*P*<0.05) (Figure 2D). The cell viability and colony formation were not significantly influenced by the transfection of INC (Figure 2C,D).

**Figure 2:** The proliferation of RA-HFLSs (**A**) The viability (OD_495_ value) of RA-HFLSs under the treatment of different concentrations of TNF-α (*n*=5); (**B**) The mRNA expression of miR-142-3p was detected by quantitative real-time PCR; (**C**) The viability of RA-HFLSs under the treatment of 10 µg/l TNF-α for different times (*n*=5). (**D**) The number of cell clones formed by TNF-α-treated RA-HFLSs (*n*=5). Mock, RA-HFLSs without treatment; TNF-α, RA-HFLSs treated with TNF-α; INC + TNF-α, RA-HFLSs transfected with miR-142-3p INC and treated with TNF-α; Inhibitor + TNF-α, RA-HFLSs transfected with miR-142-3p inhibitor and treated with TNF-α. a, b, and c, *P*<0.05 versus 0, 5, 10, 20 mg/l TNF-α, respectively (A). *, *P*<0.05 versus Mock and INC (B). *, *P*<0.05 versus Mock; #, *P*<0.05 versus TNF-α and INC + TNF-α (B and C).

### Down-regulation of miR-142-3p promoted TNF-α-induced apoptosis of RA-HFLSs

The apoptosis of RA-HFLSs was detected by TUNEL staining. As shown in Figure 3A,B, the apoptosis rate of RA-HFLSs was significantly lower in TNF-α group than in Mock group (*P*<0.05). The transfection of miR-142-3p inhibitor significantly increased the apoptosis rate of TNF-α-treated RA-HFLSs (*P*<0.05) (Figure 3A,B). In addition, the expression of B-cell lymphoma-2 (Bcl-2), an apoptotic marker was significantly higher in TNF-α group than in Mock group at both the mRNA and protein level (*P*<0.05). On the contrary, the expressions of Bax and Bad in TNF-α group were remarkedly lower than those in Mock group (*P*<0.05). The transfection of miR-142-3p inhibitor significantly down-regulated Bcl-2 and up-regulated Bax and Bad in TNF-α-treated RA-HFLSs (*P*<0.05) (Figure 3C,D). The apoptosis rate and the expressions of Bcl-2, Bax, and Bad were not significantly influenced by the transfection of INC (Figure 3A–D).

**Figure 3:** The apoptosis of RA-HFLSs (**A**) TUNEL staining of RA-HFLSs under microscope (×100); (**B**) The apoptosis rate of RA-HFLSs (*n*=5); (**C**) The relative mRNA expression of Bcl-2, Bax and Bad. (**D**) The relative protein expression of Bcl-2, Bax and Bad. Mock, RA-HFLSs without treatment; TNF-α, RA-HFLSs treated with TNF-α; INC + TNF-α, RA-HFLSs transfected with miR-142-3p INC and treated with TNF-α; Inhibitor + TNF-α, RA-HFLSs transfected with miR-142-3p inhibitor and treated with TNF-α. *, *P*<0.05 versus Mock; #, *P*<0.05 versus TNF-α and INC + TNF-α.

### Down-regulation of miR-142-3p inhibited TNF-α-induced migration and invasion of RA-HFLSs

The migration and invasion of RA-HFLSs was detected by wound healing assay and transwell assay, respectively. As shown in Figure 4A, the migration rate of RA-HFLSs was significantly higher in TNF-α group than in Mock group (*P*<0.05). The transfection of miR-142-3p inhibitor significantly decreased the migration rate of TNF-α-treated RA-HFLSs (*P*<0.05). The migration of RA-HFLSs was not significantly influenced by the transfection of INC (Figure 4A). Consistent results with the migration rate were observed on the number of invasive RA-HFLSs (Figure 4B).

**Figure 4:** The migration and invasion of RA-HFLSs (**A**) The migration rate detected by wound healing assay (*n*=5); (**B**) The number of invasive cells detected by transwell assay (*n*=5). Mock, RA-HFLSs without treatment; TNF-α, RA-HFLSs treated with TNF-α; INC + TNF-α, RA-HFLSs transfected with miR-142-3p INC and treated with TNF-α; Inhibitor + TNF-α, RA-HFLSs transfected with miR-142-3p inhibitor and treated with TNF-α. *, *P*<0.05 versus Mock; #, *P*<0.05 versus TNF-α and INC + TNF-α.

### Down-regulation of miR-142-3p inhibited TNF-α-induced inflammation of RA-HFLSs

The inflammation of RA-HFLSs was evaluated by the levels of IL-6 and MMP-3. As shown in Figure 5A,B, the contents of IL-6 and MMP-3 were significantly higher in TNF-α group than in Mock group (*P*<0.05). The transfection of miR-142-3p inhibitor significantly decreased the contents of IL-6 and MMP-3 in TNF-α-treated RA-HFLSs (*P*<0.05). The contents of IL-6 and MMP-3 were not significantly influenced by the transfection of INC (Figure 5A,B). Consistent results with the contents of IL-6 and MMP-3 were observed on the expression of IL-6 and MMP-3 in RA-HFLSs at the mRNA level (Figure 5C,D).

**Figure 5:** The levels of inflammatory factors in RA-HFLSs (**A**) IL-6 content; (**B**) MMP-3 content; (**C**) Relative IL-6 mRNA expression detected by qRT-PCR; (**D**) Relative MMP-3 mRNA expression detected by qRT-PCR. Mock, RA-HFLSs without treatment; TNF-α, RA-HFLSs treated with TNF-α; INC + TNF-α, RA-HFLSs transfected with miR-142-3p INC and treated with TNF-α; Inhibitor + TNF-α, RA-HFLSs transfected with miR-142-3p inhibitor and treated with TNF-α. *, *P*<0.05 versus Mock; #, *P*<0.05 versus TNF-α and INC + TNF-α.

### Down-regulation of miR-142-3p inhibited TNF-α-induced activation of NF-κB in RA-HFLSs

In order to reveal the regulatory mechanisms of miR-142-3p relating with NF-κB signaling, the expression of IRAK1, Toll-like receptor 4 (TLR4), NF-κB p65 and phosphorylated NF-κB p65 (p-NF-κB p65) were detected in RA-HFLSs. As shown in Figure 6, the expression of IRAK1, TLR4, and p-NF-κB p65 in RA-HFLSs were significantly higher in TNF-α group than in Mock group (*P*<0.05). The transfection of miR-142-3p inhibitor significantly decreased the expression of IRAK1, TLR4, and p-NF-κB p65 in TNF-α-treated RA-HFLSs (*P*<0.05). The expression of IRAK1, TLR4, and p-NF-κB p65 were not significantly influenced by the transfection of INC. In addition, NF-κB p65 expression was not statistically siginificant between different groups (Figure 6).

**Figure 6:** The expression of IRAK1, TLR4, NF-κB p65, and p-NF-κB p65 in RA-HFLSs detected by Western blot Mock, RA-HFLSs without treatment; TNF-α, RA-HFLSs treated with TNF-α; INC + TNF-α, RA-HFLSs transfected with miR-142-3p INC and treated with TNF-α; Inhibitor + TNF-α, RA-HFLSs transfected with miR-142-3p inhibitor and treated with TNF-α. *, *P*<0.05 versus Mock; #, *P*<0.05 versus TNF-α and INC + TNF-α.

### IRAK1 was a target of miR-142-3p

Since the miR-142-3p inhibitor significantly down-regulated IRAK1 in TNF-α-treated RA-HFLSs, the specific interaction between IRAK1 and miR-142-3p was further analyzed. As shown in Figure 7A, a binding site of miR-142-3p was predicted at 3′-UTR of IRAK1 by an online target gene prediction software (Target Scan) (Figure 7A). In addition, DLR assay showed that the fluorescence intensity was significantly lower in HEK-293T cells co-transfected with IRAK1-WT + miR-142-3p mimics than those co-transfected with IRAK1-MT + miR-142-3p mimics, IRAK1-MT + NC, and COL1A1-WT + NC (*P*<0.05) (Figure 7B).

**Figure 7:** The interaction between miR-142-3p and IRAK1 (**A**) A binding site of miR-142-3p at 3′-UTR of IRAK1 predicted by the software of Target Scan; (**B**) Relative fluorescence intensity of HEK-293T cells co-transfected with IRAK1-wild-type (WT)/IRAK1-mutant (MT) and miR-142-3p mimics (mimics)/miR-142-3p mimics NC. *, *P*<0.05 versus MT + mimics, MT + NC, and WT + NC.

## Discussion

HFLSs are key effector cells in RA, which exhibit aggressive phenotypes, such as enhanced proliferation and migration, and the overproduction of inflammatory cytokines and chemokines [27,28]. TNF-α is a proinflammatory cytokine that plays a key regulatory role in the aggressive phenotypes of RA-HFLSs. It has been reported that TNF-α promotes the proliferation, migration, invasion, and MMPs expression in RA-HFLSs [29]. TNF-α induces the proliferation of RA-HFLSs, and the production of IL-6 and IL-1β [30]. In the present study, we found that TNF-α-treated RA-HFLSs exhibited significantly increased cell viability, number of cell clones, migration rate, number of invasive cells, expression of Bcl-2, and levels of IL-6 and MMP-3, as well as decreased apoptosis rate. Our findings are just consistent with pervious studies, and further illustrate that TNF-α activates the aggressive phenotypes of RA-HFLSs.

MiR-142-3p is a specific miR that plays a dual role in tumorigenesis. miR-142-3p not only acts as a tumor suppressor in osteosarcoma [31], gastric cancer [32], colon cancer [33], and non-small-cell lung cancer [34], but also acts as a tumor promoter in pediatric brain tumor [35], renal cell carcinoma [36], and colorectal cancer [37]. Over the past decade, non-coding RNAs including miRNAs and lncRNA gradually become important regulators of inflammation [38]. Until now, the knowledge on roles of miR-142-3p on RA are still limited. In the present study, we found that the expression of miR-142-3p was significantly higher in synovial tissues and RA-HFLSs of RA patients than those of OA patients. These results are consistent with pervious studies on miR-146 [12], -155 [13], -203 [14], -221 [15], and -126 [16], and illustrate that miR-142-3p is up-regulated in RA. In addition, we also found that the expression of miR-142-3p in synovial tissues was significantly higher in RA patients at stage IV than in those at stage III. This result indicates that miR-142-3p expression may be positively associated with the severity of RA. A pervious study indicates that circulating peripheral blood miRs, including miR-16, -21, -24, -26a, -125a-5p, -125b, -126-3p, -223, and -451 are promising non-invasive biomarkers for the detection of RA [39]. We suspect that miR-142-3p may also be used as a biomarker for the diagnosis of RA.

The specific regulatory effects of miR-142-3p on the aggressive phenotypes of RA-HFLSs were further evaluated in the present study. We found that the transfection of miR-142-3p inhibitor significantly decreased the cell viability, the number of cell clones, the migration rate, the number of invasive cells, and the expression of Bcl-2 expression, and increased the expressions of Bax and Bad, and the apoptosis rate of TNF-α-treated RA-HFLSs. A pervious study has proved that the down-regulation of miR-221 inhibits the migration and invasion, and promotes the apoptosis of HFLSs [15]. Our findings are just consistent with miR-221, and illustrate that the down-regulation of miR-142-3p reverses the promoting effects of TNF-α on the proliferation, migration, and invasion of RA-HFLSs. In addition, evidences have proved that miR-142-3p is involved in the regulation of inflammatory process. For examples, miR-142-3p overexpression inhibits LPS-induced production of IL-1, IL-6, and TNF-α in articular cartilage tissues of OA mice [24]. MiR-142-3p overexpression alleviates bleomycin-induced production of IL-1 and TNF-α in MLE-12 cells [22]. In the present study, we found that the transfection of miR-142-3p inhibitor significantly decreased the contents and the expression of IL-6 and MMP-3 in TNF-α-treated RA-HFLSs. These results indicate that the down-regulation of miR-142-3p inhibits TNF-α-induced inflammation of RA-HFLSs. However, our findings are inconsistent with previous studies. Similar with the dual roles of miR-142-3p in tumorigenesis, we suspect that miR-142-3p may exert different regulatory roles on inflammation in different diseases. To sum up, the down-regulation of miR-142-3p may contribute to the amelioration of RA via relieving the aggressive phenotypes of RA-HFLSs, including the enhanced proliferation, migration, invasion, and inflammation, as well as inhibited apoptosis.

Since RA is a chronic inflammatory disease of the synovial joints, activated NF-κB is always detected in synovial tissues of RA [40]. In the present study, we found that TNF-α significantly up-regulated IRAK1, TLR4, and p-NF-κB p65 in RA-HFLSs. These results illustrate that TNF-α induces the activation of NF-κB signaling in RA-HFLSs. In RA-HFLSs, TNF-α stimulation can result in phosphorylation of NF-κB and activation of NF-κB, and then induce the expression of target genes involved in proinflammation, cell cycle, and anti-apoptosis [41]. TNF-α-induced activation of NF-κB signaling contributes to the aggressive phenotypes of RA-HFLSs. NF-κB is a common nuclear transcription factor appeared in osteoblasts. Studies have found that Runx [42], NF-κB signaling [43], and other pathways play important role in osteogenesis differentiation and activity. Cross talks between these pathways or together they regulate osteoblast activity. Disruption of Runx1 and Runx3 could result in bone marrow failure [44], and Runx3 deficiency leads to myeloproliferative disorder [45]. Changes in NF-κB pathway could regulate variations in osteogenesis activity. In the present study, the regulatory mechanisms of miR-142-3p relating with NF-κB signaling were further evaluated. We found that transfection of miR-142-3p inhibitor significantly down-regulated IRAK1, TLR4, and p-NF-κB p65 in TNF-α-treated RA-HFLSs. These results illustrate that the down-regulation of miR-142-3p inhibits TNF-α-induced activation of NF-κB signaling in RA-HFLSs. We suspect that the down-regulation of miR-142-3p may relieve the aggressive phenotypes of RA-HFLSs through inhibiting NF-κB signaling. Besides, our further assays showed that IRAK1 was a target of miR-142-3p. Since IRAK1 is partially responsible for IL1-induced activation of NF-κB signaling [46], the down-regulation of miR-142-3p may inhibit NF-κB signaling by targeting IRAK1.

In conclusion, miR-142-3p was up-regulated in RA synovial tissues and RA-HFLSs. The down-regulation of miR-142-3p significantly relieved TNF-α-induced aggressive phenotypes of RA-HFLSs, including enhanced proliferation, migration, invasion, and inflammation, as well as inhibited apoptosis. In addition, the down-regulation of miR-142-3p inhibited NF-κB signaling by targeting IRAK1, thereby contributing to the remission of TNF-α-induced aggressive phenotypes of RA-HFLSs. Down-regulation of miR-142-3p may be used as a promising therapeutic target for RA.

## Abbreviations

ANOVA: analysis of variance
Bcl-2: B-cell lymphoma-2
DLR: dual luciferase reporter gene
DMSO: dimethyl sulfoxide
FBS: fetal bovine serum
GAPDH: glyceraldehyde-3-phosphate dehydrogenase
H-DMEM: high-glucose Dulbecco’s modified Eagle medium
HEK: human embryonic kideney
HRP: horseradish peroxidase
IL: interleukin
INC: inhibitor negative control
IRAK1: IL-1 receptor-associated kinase 1
MMP-3: matrix metalloproteinase 3
MTT: 3-(4,5-dimethyl-2-thiazolyl)-2,5-diphenyl-2-H-tetrazolium bromide
NC: negative control
NF-κB: nuclear factor-κB
OA: osteoarthritis
OA-HFLS: osteoarthritis human fibroblast-like synoviocyte
OD: optical density
PBS: phosphate buffer saline
p-NF-κB p65: phosphorylated NF-κB p65
qRT-PCR: quantitative real-time PCR
RA: rheumatoid arthritis
RA-HFLS: rheumatoid arthritis human fibroblast-like synoviocyte
TBST: tris-buffered saline Tween
TLR4: toll-like receptor 4
TNF-α: tumor necrosis factor α
TUNEL: terminal dexynucleotidyl transferase-mediated dUTP nick end labeling

## References

[1] SmolenJ.S., AletahaD. and McinnesI.B. (2016) Rheumatoid arthritis. Lancet388, 2023–203810.1016/S0140-6736(16)30173-827156434

[2] ShrivastavaA.K. and PandeyA. (2013) Inflammation and rheumatoid arthritis. J. Physiol. Biochem.69, 335–34710.1007/s13105-012-0216-523385669

[3] NaqviA.A. (2017) Development of evidence-based disease education literature for pakistani rheumatoid arthritis patients. Diseases5, pii: E2710.3390/diseases5040027PMC575053829156638

[4] BurmesterG.R. and PopeJ.E. (2017) Novel treatment strategies in rheumatoid arthritis. Lancet389, 2338–234810.1016/S0140-6736(17)31491-528612748

[5] ArendW.P. and DayerJ.M. (2014) Inhibition of the production and effects of interleukins‐1 and tumor necrosis factor α in rheumatoid arthritis. Arthritis Rheum.38, 151–16010.1002/art.17803802027848304

[6] ToussirotE. and WendlingD. (2007) The use of TNF-alpha blocking agents in rheumatoid arthritis: an overview. Expert Opin. Pharmacother.8, 2089–210710.1517/14656566.8.13.208917714062

[7] CY-F. (2006) A systematic review of the effectiveness of adalimumab, etanercept and infliximab for the treatment of rheumatoid arthritis in adults and an economic evaluation of their cost-effectiveness. Health Technol. Assess. (Rockv)10, 1–22910.3310/hta1042017049139

[8] DongJ.R. (2012) Development of TNF-alpha inhibitor drugs in treatment of rheumatoid arthritis. In Int. Conf. Biomed. Eng. Biotechnol.149–152

[9] KeystoneE.C. (2011) Does anti-tumor necrosis factor-α therapy affect risk of serious infection and cancer in patients with rheumatoid arthritis?: a review of longterm dataJ. Rheumatol.38, 1552–156210.3899/jrheum.10099521572154

[10] MoulisG. (2012) Cancer risk of anti-TNF-α at recommended doses in adult rheumatoid arthritis: a meta-analysis with intention to treat and per protocol analyses. PLoS ONE7, e4899110.1371/journal.pone.004899123155441PMC3498371

[11] FurerV. (2010) The role of microRNA in rheumatoid arthritis and other autoimmune diseases. Clin. Immunol.136, 1–1510.1016/j.clim.2010.02.00520223711

[12] TomoyukiN. (2010) Expression of microRNA-146 in rheumatoid arthritis synovial tissue. Arthritis Rheum.58, 1284–129210.1002/art.23429PMC274992718438844

[13] JoannaS. (2014) Altered expression of MicroRNA in synovial fibroblasts and synovial tissue in rheumatoid arthritis. Arthritis Rheum.58, 1001–100910.1002/art.2338618383392

[14] JoannaS. (2011) Altered expression of microRNA-203 in rheumatoid arthritis synovial fibroblasts and its role in fibroblast activation. Arthritis Rheum.63, 373–38110.1002/art.3011521279994PMC3116142

[15] YangS. and YangY. (2015) Downregulation of microRNA-221 decreases migration and invasion in fibroblast-like synoviocytes in rheumatoid arthritis. Mol. Med. Rep.12, 239510.3892/mmr.2015.364225891943

[16] QuY. (2016) MicroRNA-126 affects rheumatoid arthritis synovial fibroblast proliferation and apoptosis by targeting PIK3R2 and regulating PI3K-AKT signal pathway. Oncotarget7, 74217–7422610.18632/oncotarget.1248727729613PMC5342047

[17] NiedererF. (2012) Down-regulation of microRNA-34a* in rheumatoid arthritis synovial fibroblasts promotes apoptosis resistance. Arthritis Rheum.64, 1771–177910.1002/art.3433422161761

[18] NakamachiY.MicroRNA-124a is a key regulator of proliferation and monocyte chemoattractant protein 1 secretion in fibroblast-like synoviocytes from patients with rheumatoid arthritis. Arthritis Rheum.60, 1294–130410.1002/art.2447519404929

[19] LinJ. (2014) A novel p53/microRNA-22/Cyr61 axis in synovial cells regulates inflammation in rheumatoid arthritis. Arthritis Rheum.66, 49–5910.1002/art.3814224449575

[20] RuedelA. (2015) Expression and function of microRNA-188-5p in activated rheumatoid arthritis synovial fibroblasts. Int. J. Clin. Exp. Pathol.8, 660726261542PMC4525876

[21] Reference deleted

[22] GuoF. (2017) microRNA-142-3p inhibits apoptosis and inflammation induced by bleomycin through down-regulation of Cox-2 in MLE-12 cells. Braz. J. Med. Biol. Res.50, e597410.1590/1414-431x2017597428678919PMC5496156

[23] TalebiF. (2017) MicroRNA-142 regulates inflammation and T cell differentiation in an animal model of multiple sclerosis. J. Neuroinflammation14, 5510.1186/s12974-017-0832-728302134PMC5356264

[24] WangX. (2016) MicroRNA-142-3p inhibits chondrocyte apoptosis and inflammation in osteoarthritis by targeting HMGB1. Inflammation39, 1718–172810.1007/s10753-016-0406-327447821

[25] LivakKJ and SchmittgenT.D. (2001) Analysis of relative gene expression data using real-time quantitative PCR and the 2(-Delta Delta C(T))Method. Methods25, 402–40810.1006/meth.2001.126211846609

[26] GarzonR. (2008) Distinctive microRNA signature of acute myeloid leukemia bearing cytoplasmic mutated nucleophosmin. Proc. Natl. Acad. Sci. U.S.A.105, 3945–395010.1073/pnas.080013510518308931PMC2268779

[27] LiG. (2018) SIRT1 inhibits rheumatoid arthritis fibroblast-like synoviocyte aggressiveness and inflammatory response via suppressing NF-κB pathway. Biosci. Rep.38, pii: BSR2018054110.1042/BSR20180541PMC601370629784872

[28] MaeshimaK. (2016) Abnormal PTPN11 enhancer methylation promotes rheumatoid arthritis fibroblast-like synoviocyte aggressiveness and joint inflammation. JCI Insight1, e86580, 10.1172/jci.insight.8658027275015PMC4889026

[29] ZengS. (2017) Halofuginone inhibits TNF-α-induced the migration and proliferation of fibroblast-like synoviocytes from rheumatoid arthritis patients. Int. Immunopharmacol.43, 187–19410.1016/j.intimp.2016.12.01628013187

[30] LiuN. (2017) Paeonol protects against TNF-alpha-induced proliferation and cytokine release of rheumatoid arthritis fibroblast-like synoviocytes by upregulating FOXO3 through inhibition of miR-155 expression. Inflamm. Res.66, 603–61010.1007/s00011-017-1041-728401267

[31] YangY.Q. (2014) MicroRNA-142-3p, a novel target of tumor suppressor menin, inhibits osteosarcoma cell proliferation by down-regulation of FASN. Tumour Biol.35, 10287–1029310.1007/s13277-014-2316-z25034529

[32] WangY. (2018) Downregulation of microRNA-142-3p and its tumor suppressor role in gastric cancer. Oncol. Lett.15, 8172–81802984981110.3892/ol.2018.8330PMC5962855

[33] ShenW.W. (2013) MiR-142-3p functions as a tumor suppressor by targeting CD133, ABCG2, and Lgr5 in colon cancer cells. J. Mol. Med.91, 989–100010.1007/s00109-013-1037-x23619912

[34] XiaoP. and LiuW.L. (2015) MiR-142-3p functions as a potential tumor suppressor directly targeting HMGB1 in non-small-cell lung carcinoma. Int. J. Clin. Exp. Pathol.8, 1080026617792PMC4637607

[35] LeeY.Y. (2014) MicroRNA142-3p promotes tumor-initiating and radioresistant properties in malignant pediatric brain tumors. Cell Transplant.23, 66910.3727/096368914X67836424816458

[36] LiY. (2016) Oncogenic microRNA-142-3p is associated with cellular migration, proliferation and apoptosis in renal cell carcinoma. Oncol. Lett.11, 123510.3892/ol.2015.402126893725PMC4734216

[37] XiangG. (2018) MicroRNA-142-3p promotes cellular invasion of colorectal cancer cells by activation of RAC1. Technol. Cancer Res. Treat17, 15330338187905010.1177/1533033818790508PMC606903130064309

[38] ChewC.L. (2018) Noncoding RNAs: master regulators of inflammatory signaling. Trends Mol. Med.24, 66–8410.1016/j.molmed.2017.11.00329246760

[39] ChurovA.V., OleinikE.K. and KnipM. (2015) MicroRNAs in rheumatoid arthritis: altered expression and diagnostic potential. Autoimmun. Rev.14, 1029–103710.1016/j.autrev.2015.07.00526164649

[40] Roman-BlasJ.A. and JimenezS.A. (2006) NF-κB as a potential therapeutic target in osteoarthritis and rheumatoid arthritis. Osteoarthritis Cartilage14, 839–84810.1016/j.joca.2006.04.00816730463

[41] LooG.V. and BeyaertR. (2011) Negative regulation of NF-κB and its involvement in rheumatoid arthritis. Arthritis Res. Ther.13, 221–22110.1186/ar332421639951PMC3218875

[42] HesseE. (2010) Zfp521 controls bone mass by HDAC3-dependent attenuation of Runx2 activity. J. Cell Biol.191, 1271–128310.1083/jcb.20100910721173110PMC3010073

[43] WangL. (2012) Involvement of p38MAPK/NF-κB signaling pathways in osteoblasts differentiation in response to mechanical stretch. Ann. Biomed. Eng.40, 1884–189410.1007/s10439-012-0548-x22441665

[44] WangC.Q. (2014) Disruption of Runx1 and Runx3 leads to bone marrow failure and leukemia predisposition due to transcriptional and DNA repair defects. Cell Rep.8, 767–78210.1016/j.celrep.2014.06.04625066130

[45] WangC.Q. (2013) Runx3 deficiency results in myeloproliferative disorder in aged mice. Blood122, 562–56610.1182/blood-2012-10-46061823741011

[46] LiuG., ParkY.J. and AbrahamE. (2008) Interleukin-1 receptor-associated kinase (IRAK)-1-mediated NF-kappaB activation requires cytosolic and nuclear activity. FASEB J.22, 2285–229610.1096/fj.07-10181618276832

